# Progressive Transmission of Medical Images via a Bank of Generative Adversarial Networks

**DOI:** 10.1155/2021/9917545

**Published:** 2021-04-28

**Authors:** Ching-Chun Chang, Xu Wang, Ji-Hwei Horng, Isao Echizen

**Affiliations:** ^1^National Institute of Informatics, Tokyo, Japan; ^2^Department of Information Engineering and Computer Science, Feng Chia University, Taichung 40724, Taiwan; ^3^Department of Electronic Engineering, National Quemoy University, Kinmen 89250, Taiwan

## Abstract

The healthcare sector is currently undergoing a major transformation due to the recent advances in deep learning and artificial intelligence. Despite a significant breakthrough in medical imaging and diagnosis, there are still many open issues and undeveloped applications in the healthcare domain. In particular, transmission of a large volume of medical images proves to be a challenging and time-consuming problem, and yet no prior studies have investigated the use of deep neural networks towards this task. The purpose of this paper is to introduce and develop a deep-learning approach for the efficient transmission of medical images, with a particular interest in the progressive coding of bit-planes. We establish a connection between bit-plane synthesis and image-to-image translation and propose a two-step pipeline for progressive image transmission. First, a bank of generative adversarial networks is trained for predicting bit-planes in a top-down manner, and then prediction residuals are encoded with a tailored adaptive lossless compression algorithm. Experimental results validate the effectiveness of the network bank for generating an accurate low-order bit-plane from high-order bit-planes and demonstrate an advantage of the tailored compression algorithm over conventional arithmetic coding for this special type of prediction residuals in terms of compression ratio.

## 1. Introduction

With the development of digital imaging equipment, more and more medical images have been produced and a medical image dataset usually contains a large number of images. Transmission of abundant medical images over a low narrow bandwidth public network will no doubt cause critical network pressure and further delay the timing of diagnosis [1].

To increase the speed of medical image transmission, some schemes have been proposed to build up more effective special networks. For instance, in [2], a unique pair of interfaces was proposed to provide a fast thoroughfare for medical data transmission between two DICOM applications and could speed up 1.22 and 13 times, respectively, in the local area networks (LAN) and wide area networks (WAN). Later, they further proposed an improved network [3] to combine the local area network (LAN) and wide area network (WAN) and used parallel TCP connections to optimize the DICOM protocol. This network can speed up about 2.2 to 3.5 times when transmitting magnetic resonance images.

On the other aspect, some new image transmission techniques have been proposed. An intuitive way is to reduce the resolution of medical images before transmission in a poor bandwidth network. However, doctors suffer from misdiagnosis with the lower resolution medical images. Therefore, the progressive image transmission (PIT) [4] technique emerges as the times require. The conventional raster scan ordered pixel by pixel image transmission technique is inefficient, and the key region of the image which indicates the disease may be received at the end of the transmission makes doctors out of patience and affects the treatment. The progressive image transmission technique usually transmits a lower resolution image at first and gradually transmits the details of the image to further increase the resolution until the original image is totally transmitted. Through the transmission, receivers can decide whether they want to receive the details of the image or not in a short time. As a consequence, doctors can control the final image resolution and the required storage space. Over the past decades, some mature PIT techniques have been proposed. The bit-plane progressive image transmission method (BPM) [5, 6] is one of the low computational complexity and intuitive technique to transmit the image bit-plane by bit-plane which is detailed in Section 2. Another sort of progressive image transmission techniques is that, in [7–12], the image is divided into nonoverlapping blocks, and a quantized pixel value is used to represent the whole block, then, progressively dividing the image into finer blocks to improve the image resolution. Some schemes [13–17] transform the image into a wavelet domain and transmit the coefficients instead of pixels. Lossy compression [18] and lossless compression [19] methods are also adopted in some schemes to reduce the file size in each round of transmission.

The deep learning technique has matured in recent years and drawn massive research which is widely used in industry [20]. Some advanced deep learning architectures have also been introduced into medical image processing. Medical image classification is the most important area where deep learning makes a great contribution. The CNN network has been widely used in medical image classification and achieved a higher accuracy [21–23]. The deep learning technique is also suitable for medical image detection. The methods for organ, region, and landmark localization [24–26] and object and lesion detection [27–29] all adopt the deep learning architectures. Then, the medical image segmentation is naturally developed in the detected images [30–32]. The other tasks on medical images processing such as content-based image retrieval [33]; image generation and enhancement [34]; and description of medical images with shape, margin, and density [35] have also been proposed. Recently, the deep learning architecture with adversarial learning: generative adversarial network (GAN) has been proposed by Goodfellow et al. [36] that has the ability to generate realistic-looking images. Based on the GAN network, a powerful architecture pix2pix [37] was set up as an image bit-plane predictor to translate the image styles and has been adopted in different scenarios such as steganography [38] and even in medical images [39, 40]. However, so far, these deep learning techniques have not been applied to the medical image transmission. By leveraging the prediction ability of the GAN network, the medical images can be compressed before transmission and thus the efficiency of transmission can be improved.

In this paper, we adopt the framework of the bit-plane PIT method to transmit medical images. To reduce the amount of data before transmission, a GAN-based predictor bank is designed to predict the bit-planes. By progressively predicting the bit-plane to be sent based on previously transmitted bit-planes, we need only to send the residual provided that the receiver can execute the same prediction. The proposed GAN-based predictor bank produces a prediction of high accuracy so that the residual can be efficiently compressed before transmission. Thus, the efficiency of bit-plane PIT is greatly improved, and the transmission cost can be reduced. The main contributions of our scheme are summarized as follows:

1. Introduce a deep neural network of pix2pix GAN network into the research of progressive medical image prediction and transmission
2. Design a GAN-based predictor bank to help bit-plane compression of medical images
3. Propose an adaptive residual bit-plane compression technique of high compression ratio

Experimental results validate the effectiveness and efficiency of the proposed prediction network and compression technique. The rest of this paper is organized as follows.  Section 2 briefly introduces the bit-plane method of the progressive image transmission.  Section 3 details the proposed adversarial learning for progressive bit-plane prediction scheme and the adaptive residual bit-plane compression technique.  Section 4 provides the experimental results to demonstrate the accuracy of our prediction scheme and the efficiency of the proposed compression technique. In addition, the performance of the proposed residual bit-plane compression is compared with the conventional arithmetic coding. The conclusions are offered in Section 5.

## 2. Bit-Plane Method of PIT

In this section, the bit-plane method of progressive image transmission (BPM) technique which has been widely used to transmit a large volume of high-resolution medical images, is briefly introduced. The progressive image transmission (PIT) technique is an effective way to transmit images over narrow bandwidth channels. Among the PIT techniques, BPM is a simple and intuitive way of transmission, which divides an image into bit-planes and sends it plane by plane. For the grayscale images, each pixel is valued from 0 to 255, that is, 256 gray levels, and can be represented by 8 bits. The original image can be decomposed into eight bit-planes from the most significant bit-plane *b*_8_ to the least significant bit-plane *b*_1_, so that *b*_8_ records the main content and *b*_1_ records the subtle details, respectively, of the original image. Therefore, in the bit-plane PIT method, bit-planes from *b*_8_ to *b*_1_ are sequentially transmitted and the receiver can progressively recover the image until all bit-planes are sent or the current image quality is satisfied. The detailed BPM method is described below.

In the most significant bit-plane *b*_8_, the bit “0” and “1” indicate the corresponding pixels are ranging from “0 to 127” and “128 to 255,” respectively. Therefore, after receiving *b*_8_, the mean values of these two intervals, that is, 64 and 192, are used to coarsely represent them. When receiving the next bit-plane *b*_7_, the receiver updates the image by using finer quantization levels of (32, 96, 160, 224) to represent corresponding codes “00,” “01,” “10,” and “11.” This process proceeds until all of the eight bit-planes are sent. An example of BPM transmission is illustrated in Figure 1, where the progressive combination of bit-planes and their corresponding recovered images are presented. As the number of received bit-planes increases, the available quantization levels also increase and a finer recovered image can be obtained.

## 3. Progressive Bit-Plane Prediction and Compression

Based on BPM progressive image transmission, we propose a bit-plane prediction method and a compression technique to improve the transmission efficiency of medical images. In this section, the proposed image transmission scheme and a pix2pix model-based bit-plane prediction method are introduced first. Then, a new technique for compression of the prediction error bit-plane is presented.

### 3.1. Adversarial Learning for Progressive Bit-Plane Prediction

For the purpose of progressively predicting image bit-plane by bit-plane, the generative adversarial network is introduced in this paper to predict and synthesize bit-planes. GAN architecture is a classical neural network to generate synthetic images of a specific style through training. The pix2pix model is a famous model of a GAN-based network which can be exploited to make an image-to-image translation. In the pix2pix model, the generator *G* is a U-Net, which is designed for biomedical image segmentation, instead of the conventional encoder-decoder net. The U-Net consists of a contracting path to downsample the input image, and an expansive path to generate an output image of full resolution. The contracting path consists of four steps connected by 2x2 max pooling layer with stride 2; each step contains three repeated 3 × 3 convolutions with ReLU. The expansive path also consists of four steps connected by 2 × 2 upconvolution and halves of the feature maps are cropped from the contracting path. For the discriminator, the PatchGAN is adopted to discriminate that the overlapping patches in the generated image are real or fake. Different from the conventional GAN discriminator which only output one result, that is, real or fake, PatchGAN outputs a matrix and each element reflects the pixel differences of the current patch between the synthetic image and the original image in the current patch region. Additionally, to obtain a generated image with higher similarity to the input original image, the Manhattan distance (*ℓ*_1_ norm) which is more suitable for high dimensional images is chosen to evaluate the difference between input and output images. Therefore, in the pix2pix model, assume *x* and *y* are the input and output images; the difference between input and output is evaluated by

(1) $$\begin{array}{c} {ℒ}_{L1}\left(G\right)=E\left[{\left\|y-G\left(x\right)\right\|}_{1}\right]. \end{array}$$

Then, the final objective is obtained by mixing the *ℓ*_1_ loss with the traditional GAN loss by

(2) $$\begin{array}{c} G^{*}=\arg\underset{G}{\min}\underset{D}{\max}{ℒ}_{\text{GAN}}\left(G,\;D\right)\;+\;\lambda {ℒ}_{L1}\left(G\right),\\ {ℒ}_{\text{GAN}}\left(G,\;D\right)=E\left[\text{log }D\left(y\right)\right]+E\left[\text{log}\left(1-D\left(G\left(x\right)\right)\right)\right], \end{array}$$

where *λ* is a hyperparameter to balance two losses to achieve better performances.

Through the above architecture, the pix2pix model can translate the input image into different styles such as color images, day-to-night, and image inpainting. Inspired by pix2pix image-to-image translation model, in this paper, we train the pix2pix model to predict bit-planes of medical images. The proposed scheme is based on the BPM of progressive image transmission. A medical image is divided into eight bit-planes and transmitted plane by plane. On the receiver side, bit-planes are also received plane by plane and the medical image can be progressively reconstructed. During transmission, we leverage the pix2pix model to generate a predicted version of the bit-plane to be sent based on the previous bit-planes. Benefiting from the high accuracy of prediction, the prediction error of bit-plane (residual bit-plane) can be compressed efficiently. Thus, a bit-plane can be transmitted by sending its residual instead. The predictors of different layers of bit-plane are trained separately, organized into a predictor bank, and shared with the receiver. When receiving the residual, the receiver can do the same prediction to obtain the predicted bit-plane, and then, the original bit-plane can be recovered according to the received residual bit-plane and the predicted bit-plane. The framework of our proposed progressive medical image transmission scheme is shown in Figure 2.

In detail, assuming the bit-planes from the MSB to LSB are *b*_8_ to *b*_1_, we feed all *b*_8_ bit-planes of training images into the model as the input images to generate output images and set their corresponding *b*_7_ bit-planes as the ground truth images. The standard format of input and output for the pix2pix model is an image of 8-bit depth. To fit this format, zeros are appended behind the provided bit-planes. When training the model for predicting *b*_6_, *b*_8_ and *b*_7_ are concatenated as the input. An illustration for this case is shown in Figure 3. The detailed prediction models for the remaining bit-planes are trained in a similar manner. Then, a series of pretrained predictors are organized into a predictor bank as shown in Figure 4, which contains seven predictors for predicting bit-planes of different layers. For instance, the *b*_6_ predictor can predict bit-plane *b*_6_ by using the bit-planes *b*_8_ and *b*_7_. Therefore, each bit-plane from *b*_7_ to *b*_1_ can be progressively predicted by its previous bit-planes. On the application phase, the residual bit-plane can be calculated by comparing the bit-plane to be sent and the synthetic one by

(3) $$\begin{array}{c} {ℛ}_{i,j}=\left\{\begin{array}{cc} 0, & \text{if }{ℬ}_{i,j}=S_{i,j},\\ 1, & \text{if }{ℬ}_{i,j}\neq S_{i,j}, \end{array}\right) \end{array}$$

where ℛ, ℬ, and *𝒮* represent the residual, original, and synthetic bit-planes, respectively. Assuming the image is sized *M* × *M*, *i*,  *j* denote the coordinates and range from 1 to *M*. In this paper, the seven residual bit-planes are denoted by symbols *r*_7_ to *r*_1_. On the receiver side, the predicted bit-plane can be obtained by the preshared predictor bank. After receiving the residual bit-plane, the real bit-plane can be recovered by

(4) $$\begin{array}{c} {ℬ}_{i,j}=\left\{\begin{array}{cc} S_{i,j}, & \text{if }{ℛ}_{i,j}=0,\\ \bar{S_{i,j}}, & \text{if }{ℛ}_{i,j}=1, \end{array}\right) \end{array}$$

where $\bar{{𝒮}_{i,j}}$ denotes the binary bit-flipped value of *𝒮*_*i*,*j*_, that is, change “1” to “0” or change “0” to “1.”

### 3.2. Adaptive Residual Bit-Plane Compression

The size of the prediction residual and its original bit-plane is the same. The major difference is that the values in the residual bit-plane are mostly zero. So, it can be compressed more efficiently. In addition, the error bits of our GAN-based bit-plane prediction are highly concentrated in the vicinity of image edges or complex details. According to the features of the residual bit-planes, we further propose an adaptive compression technique to reduce the data size. The detailed procedures are as follows:

  Step 1: decompose a residual bit-plane ℛ sized *M* × *M* into *M*^2^/*m*^2^ nonoverlapping blocks ℛ^*n*^ sized *m* × *m*, where *n* ranges from 1 to *M*^2^/*m*^2^.
  Step 2: initialize a location map *L* with the length of *M*^2^/*m*^2^.
  Step 3: scan the residual blocks in the raster scan order. If values in the block ℛ^*n*^ are all “0” or all “1,” go to Step 4; otherwise, go to Step 5.
  Step 4: set the *n*-th bit *L*^*n*^ of the location map *L* to “0,” and record the block value by one bit, that is, *z*^*n*^={*b*}, where *z*^*n*^ denotes the *n*-th segment of the recovery sequence and *b* is the common value of the block's elements.
  Step 5: set *L*^*n*^ to “1,” and record all *m*^2^ bits of the current residual block into the recovery sequence *r*^*n*^ in raster scan order.
  Step 6: return to Step 3 until all blocks have been scanned to obtain the location map *L* and the recovery sequence *r*.
  Step 7: compress the location map *L* by arithmetic coding to acquire the final location map *L*′. Then, the final compressed residual bit-plane is obtained by concatenating *L*′ and *r*.

When receiving the compressed residual bit-plane, the initial residual bit-plane can be obtained by the following decompression procedures:

  Step 1: decompress the location map *L*′ by arithmetic decoding to obtain the *M*^2^/*m*^2^ sized location map *L*.
  Step 2: if *L*^*n*^ is “0,” all bits in the current block ℛ^*n*^ are the same and go to Step 3; otherwise, go to Step 4.
  Step 3: extract one-bit *z*^*n*^ from the recovery sequence *r* and set all *m*^2^ bits in ℛ^*n*^ to *r*^*n*^.
  Step 4: extract *m*^2^ bits *z*^*n*^ from *r* and rearrange these bits in the raster scan order to recover ℛ^*n*^.
  Step 5: return to Step 2 until all blocks have been scanned. Then, the initial residual bit-plane ℛ can be obtained by tiling the recovered residual blocks in the raster scan order.

A simple example is given in Figure 5. In this example, the block size *m* is set to 2. Since the first, third, and fourth blocks are uniform valued blocks, the corresponding bits in the location map are set to 0. Meanwhile, just one sample bit is recorded into the recovery sequence for each of them. For the rest blocks, their corresponding bits in the location map are set to 1 and all bit values are recorded. When recovering these blocks, referring to the location map and the recovery sequence, all blocks can be totally recovered.

## 4. Experimental Results

In this section, we evaluate the performance of our proposed bit-plane prediction scheme with generative adversarial networks and compare our proposed residual bit-plane compression scheme with the conventional arithmetic coding compression technique. The dataset used for training and testing, the training details, and the evaluation metrics are first introduced, and then, the performance of the proposed scheme is evaluated.

### 4.1. Dataset and Training Details

The image samples for training and testing are the greyscale chest X-ray images collected from the National Institutes of Health under the U.S. Department of Health and Human Services. In our experiments, 10,000 images from the first compressed file are used for training, and the other 10 images from the fifth compressed file as shown in Figure 6 are used for performance evaluating and analyzing. Before training and testing, all the images are first downsampled into 256 × 256 sized images to fit our proposed network architecture.

When training the proposed model, each bit-plane prediction is trained over 100 epochs and the initial learning rate and the batch size are set to 2 × 10^−4^ and 32, respectively. The learning rate is enforced halfway during training and the hyperparameter *λ* is set to 10^3^. The model parameters are updated and optimized by the Adam function.

### 4.2. Evaluation Metrics

To evaluate the performance of the predicted bit-planes, two important metrics, error rate (ER) and the compression ratio (CR), are introduced in this paper to conduct some experiments. For a predicted bit-plane, referring to its original bit-plane, if the two bits in the same place are the same, the corresponding bit in the residual bit-plane is set to “0” and set to “1” when the predicted bit is incorrect. The error rate (ER) is defined as the ratio of “1's” in the residual bit-plane and can be calculated by

(5) $$\begin{array}{c} \text{ER}=\frac{\varepsilon }{M\times M}\left(\%\right), \end{array}$$

where *ε* denotes the number of error bits. After obtaining the residual bit-plane, different compression techniques are adopted to compress it. The compression ratio (CR) denotes the ratio between the data sizes of the original and the compressed versions that can be calculated by

(6) $$\begin{array}{c} \text{CR}=\frac{M\times M}{\delta }, \end{array}$$

where *δ* represents the data size, in bits, of the compressed residual. Generally, the compression ratio is greatly dependent on the error rate, and a residual of a low error rate can be compressed more efficiently. Thus, a prediction of high accuracy can improve the transmission efficiency.

### 4.3. Performances

First, the test image “Image 05” is used to demonstrate the experimental results of the original bit-planes, prediction bit-planes, and corresponding residual bit-planes.

From Figure 7, when receiving the bit-plane 8, the rest bit-planes can be progressively synthesized to obtain the predicted bit-planes. In the residual bit-plane, the white pixels are the error predictions, and most of them are concentrated in the edges of the image. The error rate of the bit-plane 7 is the lowest because this bit-plane is relatively smooth and just a few edges are presented. The error rate gradually increases as the details of a bit-plane become more complex. Nevertheless, the error rate of bit-plane 1 is still lower than 35% and most bits can be accurately predicted. Therefore, the proposed scheme can progressively predict bit-planes with high accuracy. To further verify the prediction accuracy, Table 1 lists all error rates of different layers in ten test images.

The error rate monotonously increases from *r*_7_ to *r*_1_. Two exceptions occur in “Image 04” and “Image 06”: the error rate of *r*_6_ is lower than *r*_7_. The lowest error rate and highest error rate are 5.9723% and 36.1099%, respectively, in *r*_7_ of “Image 07” and *r*_1_ of “Image 09.” Generally, the average error rate monotonously increases from high bit-plane to low bit-plane. The average error rate for an entire image is 19.2673%.

The compression ratio is greatly dependent on the error rate and the distribution of error bits. A residual bit-plane with a few concentrated error bits can be compressed efficiently. The compression ratio of the residual bit-planes is plotted in Figure 8. Since the number of error bits increases from *r*_7_ to *r*_1_, the compression ratio decreases as the bit layer decreases. Even in the exception cases of “Image 04” and “Image 06,” where the error bits of *r*_7_ are more than *r*_6_, the compression ratio of *r*_7_ is also greater due to the concentrated distribution of error bits.

To investigate the effect of block size setting, four different sizes are applied to compress the residual. The compression ratio for different block sizes and bit layers is listed in Table 2. The compression ratio of size 4 is significantly greater than the other sizes for all layers of bit-planes.

Additionally, our proposed residual bit-plane compression technique is also compared with the arithmetic coding technique. As shown in Figure 9, the average compression ratio of our proposed scheme is significantly better in the bit-planes of *r*_7_ and *r*_6_, while the performance of arithmetic coding is slightly better in the bit-planes of *r*_4_ and *r*_3_. That is because, in the rear residual bit-planes such as *r*_4_ to *r*_1_, the errors have no continuous distribution to make our compression technique not efficient. For compression of an entire image, the proposed scheme is significantly better than the arithmetic coding. To further verify the applicability in the medical image domain, the compression ratio for all test images is listed in Table 3. In Table 3, ℛ and ℬ denote that the sources of compression are residuals and original bit-planes, respectively. Additionally, since the original first bit-plane should be transmitted at the beginning, in two types of bit-plane ℛ and ℬ, the original first bit-plane is transmitted and compressed by different compression methods. As shown in Table 3, the compression ratio of residual is greater than that of the original version. It implies the devised GAN predictor bank is helpful. In addition, the proposed bit-plane compression technique outperforms the arithmetic coding in the scheme of bit-planewise compression. As shown in the experimental results, the compression ratio is severely affected by the smoothness of residual bit-planes. In medical images, most of the textures are concentrated in the region of interest, which is particularly suitable for the proposed predictor bank to work efficiently. Additionally, the parameters of the pretrained predictor bank are crucial for the sender and receiver, so that the predictor bank needs to be protected to ensure applicability and security.

## 5. Conclusions

In this paper, we introduce a GAN predictor bank and a bit-plane compression technique into the progressive transmission of medical images. Experimental results validate the proposed predictor bank can effectively predict bit-planes under the progressive scheme. Furthermore, the proposed adaptive bit-plane compression is more efficient than the arithmetic coding for the current application. This paper intends to introduce deep learning techniques into the classical progressive image transmission and we hope this paper can give some illuminations for future research. In our future works, we will further introduce and improve more convolutional neural networks into the compression and transmission of medical images.

## Figures and Tables

**Figure 1:** An illustration of the bit-plane PIT method.

**Figure 2:** The framework of our proposed scheme.

**Figure 3:** The training workflow of the network architecture.

**Figure 4:** The predictor bank for bit-plane prediction.

**Figure 5:** An example of the proposed adaptive residual bit-plane compression.

**Figure 6:** Ten test images: (a) Image 01, (b) Image 02, (c) Image 03, (d) Image 04, (e) Image 05, (f) Image 06, (g) Image 07, (h) Image 08, (i) Image 09, and (j) Image 10.

**Figure 7:** The original bit-planes (first row), the prediction bit-planes (second row), and the corresponding residual bit-planes with error rates (third row) of the test image “Image 05” (top-left).

**Figure 8:** Compression ratio of each bit-plane in ten test images when the block sizes are (a) *m*=2, (b) *m*=4, (c) *m*=8, and (d) *m*=16.

**Figure 9:** Average compression ratio comparison in each bit-plane.

**Table 1:** Error rates ER of residual bit-planes 7-1 in test images.

Images	*r*_7_	*r*_6_	*r*_5_	*r*_4_	*r*_3_	*r*_2_	*r*_1_	Average
Image 01	10.4553	12.5137	14.1861	17.9123	22.0245	26.9897	34.8251	19.8438
Image 02	11.8851	14.6881	15.9241	18.6523	21.9116	25.9674	31.4346	20.0662
Image 03	8.4518	10.7819	12.5763	18.4158	21.4813	24.8047	31.7764	18.3269
Image 04	13.2202	11.4502	14.5264	18.1915	21.5698	26.7654	34.0698	19.9705
Image 05	9.5856	10.9573	13.7833	19.2261	26.5549	24.6841	33.3908	19.7403
Image 06	10.2814	9.4879	13.6139	22.3846	22.3145	26.4420	33.3206	19.6921
Image 07	5.9723	9.6817	14.3890	16.8106	20.3964	25.3586	31.3263	17.7050
Image 08	11.3373	11.6348	12.8296	16.2766	19.9966	24.0417	31.6544	18.2530
Image 09	16.1194	12.0071	14.6622	17.5919	21.8216	27.3041	36.1099	20.8023
Image 10	10.5713	12.0087	13.3682	16.1804	20.0516	24.5636	31.1661	18.2728
Average	10.7880	11.5211	13.9859	18.1642	21.8123	25.6921	32.9074	19.2673

**Table 2:** Average bit-plane compression ratio (CR) for different block sizes.

Block size	*r*_7_	*r*_6_	*r*_5_	*r*_4_	*r*_3_	*r*_2_	*r*_1_
2	2.1295	1.8124	1.5112	1.2814	1.1327	1.0449	0.9922
4	**2.9095**	**2.2059**	**1.7053**	**1.3731**	**1.2614**	**1.2137**	**1.1426**
8	2.1585	1.5553	1.2788	1.1166	1.0435	1.0313	1.0147
16	1.4372	1.1383	1.0775	1.0266	1.0036	1.0072	1.0027

**Table 3:** Comparison of compression ratio for ten test images.

	Image 01		Image 02		Image 03		Image 04		Image 05	
	ℛ	ℬ	ℛ	ℬ	ℛ	ℬ	ℛ	ℬ	ℛ	ℬ
Proposed	1.3923	1.2352	1.4347	1.3180	1.4566	1.3087	1.3970	1.2453	1.4272	1.2650
Arithmetic coding	1.3739	1.0062	1.3475	1.0098	1.4255	1.0020	1.3629	1.0022	1.3783	1.0101

	Image 06		Image 07		Image 08		Image 09		Image 10	
	ℛ	ℬ	ℛ	ℬ	ℛ	ℬ	ℛ	ℬ	ℛ	ℬ

Proposed	1.4003	1.2409	1.4609	1.2722	1.4615	1.2953	1.3917	1.2376	1.4601	1.2835
Arithmetic coding	1.3827	1.0052	1.4585	1.0051	1.4166	1.0006	1.3349	1.0055	1.4158	1.0116

## Data Availability

The data used to support the findings of the study are available from the corresponding author upon request.
